The article "Research and Design of Docker Technology Based Authority Management System" was retracted in 2023. Reasons: unreliable results or conclusions; concerns about the data; concerns about the peer review; concerns about the citations.

# Research and Design of Docker Technology Based Authority Management System

**DOI:** 10.1155/2022/5325694

**Published:** 2022-04-13

**Authors:** Li You, Hui Sun

**Affiliations:** ^1^Information Center, Hebei Vocational University of Industry and Technology, Shijiazhuang, China; ^2^Department of Automotive Engineering, Hebei Vocational University of Industry and Technology, Shijiazhuang, China

## Abstract

With the development of mobile Internet technology and the continuous popularization of the network, various kinds of network software come out constantly and people are becoming more and more dependent on them, while role authority management is of great importance for the security of software, the control of management process, and the usability of users. In terms of system implementation, virtual machine technology is often faced with problems such as high virtualization overhead, poor scalability, and long deployment time in spite of its good isolation effect. Container technology represented by Docker can well solve these problems and make it possible to quickly build, deploy, operate, and maintain as well as expand services. Based on Docker technology, this research compares and chooses from various authority control models and finally decides to take the role authority management model as the infrastructure. It designs the role authority control model based on cloud computing and Docker technology in combination with the Task Controller Function, the Project Controller Function, and the User Controller Function and realizes this model by adopting the MongoDB database combined with HTML/CSS/Javascript syntax and the Boor Strap framework. After the test, it is found that the Docker technology based role authority management system has satisfactory test performance consistent with expected outputs as well as strong robustness, which can meet the requirements of different objects and subjects.

In the era of data nowadays, role authority management is no longer limited by region or system but is gradually applied to all kinds of systems and has become one of their important components. Role authority management is applied in various systems with the purpose that the module can control and manage the system authorities [1–5]. System management authorities, if not rationally and effectively controlled and managed, will bring about system bugs, information leakages, and other problems that cause serious loss of users [6–10]. Therefore, in order to avoid such problems, it is of great necessity to strengthen the control and management of system authorities. This paper studies the design and realization of the role authority management system based on the cloud computing platform and obtains the implementation interface of the role authority management system based on the cloud computing platform, which enhance the robustness of role authority management system design and development and lower risks.

## 1. Research Status

With the development of mobile Internet technology and the continuous popularization of the network, various kinds of Web software come out in the sight of the public one after another. As the most commonly used function in Web systems, user role authority management is constantly studied.

Research on user role authority in software systems began in 1996 when Professor Ravi Sandhu et al. proposed the RBAC (Role-Based Access Control) model [11], where the concept of user role is introduced for the first time. At present, there are discretionary access control models, mandatory access control models, and role-based access control models. As cloud computing technology and distributed storage technology develop rapidly with the advent of the big data era, data security has become the focus of people's attention, and the access control of cloud systems has become an urgent problem to be solved. In order to improve the security of traditional access control technology, constraint research based on role access control has become a research hotspot nowadays.

In 1997, Professor Ravi Sandhu proposed the ARBAC97 model (distributed RBAC management model) [12]. On the basis of these two models, the ARBAC99 model and the ARBAC02 model [13] improved the management function of RBAC. After the RBAC96 model, another famous RBAC model is the RBAC2001 model [14] proposed by the American National Institute of Standards and Technology. Up to now, RBAC is still a topic concerned and studied by relevant scholars. According to the relevant research of Mohsen Saffarian et al., they organically integrated DAC and RBAC model to construct the OB-RBAC model. This model can be more applicable to the settings of organizations with higher flexibility or those with lack of standardization. However, when authorities and users increase gradually, this authorization management method will become highly complicated [15, 16].

In China, researchers mainly put forward improvements to the RBAC model in specific practical studies. In order to strengthen the further management of user roles in the system, Fan et al. proposed a role management method based on the RBAC model in 2012 [17]. Zhang et al. proposed a dynamic role access control model based on attribute value variation in 2016 by setting attributes for roles [18], thus realizing the conversion between dynamic roles and static roles. On the basis of retaining the easy authorization and hierarchical management of roles of the RBAC model and in view of the SaaS (Software-as-a-Service) [19] multitenant mode, Xiong et al. proposed a multitenant, multidomain, and secure interoperation access control method based on the role-level tree [20]. In view of the limitations and complementarity of RBAC and ABAC (Attribute-Based Access Control) in large-scale environments, Zhou and Ren proposed an access control model combining attributes and roles in 2018. On this basis, the existing models are divided into three types: dynamic role models, attribute-centered models, and role-centered models [21].

Through the analysis of research status, problems such as low execution efficiency, unbalanced distribution of resources, and complex deployment process are found in the studies abovementioned. Docker provides great convenience to developers with not only standard container specification technology and image specification but also a series of user-friendly container management platforms. It quickly takes up a large market share and many systems have been deployed on Docker. Therefore, this paper employs the operation layer to realize the interaction of front page data, makes advantage of the related methods in the Dao layer to process background data, takes Docker technology as the basis for designing the technical framework, and combines the Task Controller Function, the Project Controller Function, and the User Controller Function to meet the requirements of different objects and subjects. The research idea and the model and framework designed also become the innovation point of this paper.

## 2. Overview of Docker Technology

In cloud computing, PaaS (Platform as a Service) is a service mode that can provide users with software platforms and development environments [22–25]. Docker is an open-source project realized on the basis of Golang and the application of Docker can accelerate the realization of PaaS mode [26]. In software development, we usually encounter software reuse failures caused by development environment difference, while Docker can effectively solve such problems. Whether during the development stage or test stage of software, Docker can create the same environment. In other words, it intervenes in the container configuration to guarantee the consistency of the dependence of all configurations within the container and to enable that the development, test, and release of software all occur in the same environment. Docker has three advantages. First, it can use the image repository. Second, it can conduct continuous deployment test. Third, it possesses high level of resource utilization. In this paper, the role-based authority management system is deployed on the Docker platform. After the server is started and the images are obtained, the installation of operating systems, repositories, and application services will be completed, which greatly shortens the system development process. Just because Docker does not need to start the slave operating system, enough disk space is spared, abundant system resources are saved, and the utilization rate of system resources is improved. It can also be considered that the virtualization of virtual machines is manifested in hardware level and the virtualization of Docker is manifested in operating system level. The architecture of Docker is as shown in Figure 1.

It can be seen in Figure 1 that the Server Docker is the kernel daemon which can be deployed not only locally but also in remote servers. The communication bridge between Server and Client is Rest APL. As the Client, Client Docker CL1 can, besides providing corresponding interfaces for users, manage containers and images. After images are packaged, users can create containers by virtue of images and then operate them, during which Server can be invoked to control disk resources. Compose in Docker is employed to conduct rapid arrangement of container clusters before the operation of multiple containers. Practically, it is hard to provide sound operating conditions for the system by relying on only one single container, and the database and server need to be started simultaneously to guarantee the sound system operation. Besides, service and project are two important concepts in Compose. The first means that it can define the services required by the application in terms of the name, network, configuration environment, dependence condition, etc. Service is conducted in the granularity of container and each container carries one service. The second refers to the whole project that needs to be implemented by users. The content (container deployment, container management, etc.) disclosed in YMAL file can be deemed as a project and Compose will usually manage the project without extra interference.

## 3. Model Building and Design of Background Authority Functions

### 3.1. Basic Model Building

Build the authority management system model on the basis of the role-based access control technology. Due to the large scale of the system, we can not conduct authority setting and role division for every user in traditional ways. The concept of user group should be introduced and users with the same authorities and characteristics should be divided into the same user group without changing the many-to-many relationship in role-based access control. One user can be divided into multiple user groups and one user group relates to multiple users. This can not only reduce the heavy and complicated workload but also facilitate subsequent management. Take the task management system as an example. Users can be divided into two user groups: first, the project participant user group, and second, the project administrator user group. Different user groups have different authorities. For example, roles in the administrator user group have authorities to modify and delete the project while roles in the participant user group only have authorities to preview and edit the tasks but cannot modify or delete the project. See Figure 2.

### 3.2. Comparison and Option of Authority Control Models

In user information management systems, authority control is one necessary link. The so-called authority means that users need to access authorized content in accordance with the security rules set by the system. Authority control can effectively identify user identity and avoid illegal invasion; therefore, authority control has been widely promoted in numerous user login systems. Current authority control technologies can fall into two categories: the system level security management, such as operating system level security management and database level authority management, etc., and the application-level security management which generally is closely related to specific system requirements. From the perspective of implementation, authority control mainly employs three types of models: (1) the discretionary access control model; (2) the mandatory access control model; and (3) the role-based access control model.

#### 3.2.1. Discretionary Access Control

It means that the subject with control power can authorize the access right of the object to other subjects [27]. In such access management model, one user can have different authorities to different resource objects while different users can have different authorities to one same resource object; one user can authorize his authority to other users without any limitation. In the discretionary access control model, users can formulate corresponding protection strategies for the resource object to be protected according to system requirements. Discretionary access control has advantages such as flexible authority distribution, simple and easy-to-use models, and strong expansibility; however, the discretionary pattern of authorization leads to low security level of the whole system while the high complexity of discretionary authorization is also a hard nut to crack.

#### 3.2.2. Mandatory Access Control

Its main function is to prevent virus attacks and ensure the confidentiality and security of information [28]. The access control method is to mark the security of the elements in the system, that is, to give each subject (user, process) and object (file, data) a security level and restrict the access behavior of the subject to the object by comparing their different security levels. In the mandatory access control model, access control is executed mandatorily by the system and users do not have authority to change their security level. The most typical mandatory access control model is the Bell-LaPadula model, the relevant access control rules of which are as shown in Table 1.

It can be seen in Table 1 that there are four security levels for objects and subjects which are A (top-secret), B (secret), C (confidential), and D (unclassified) successively from top to bottom. Read and write operations are represented by I and Q in Table 1, respectively. The access control rules are as follows: (1) when the security level of the subject is higher than that of the object, the subject can execute the read operation to the object; (2) when the security level of the subject is lower than that of the object, the subject can execute the write operation to the object. Such feature is usually called “Read Down, Write Up.” Such access rules can effectively prevent subjects of lower security level from accessing resources of higher security level, which guarantees information confidentiality.

#### 3.2.3. Role-Based Access Control

Such model successfully integrates the concept of role into users and authorities [29–31]. Users can play their required part of roles in a reasonable scope and all roles have their authorities and then work accordingly. The core structure of this model is as shown in Figure 3.

In this model, users and authorities are not completely corresponding for one user can play the part of multiple roles and one role can have multiple users on the contrary. As well, the relation between roles and authorities is not single but has many-to-many characteristics. The relation of the three is as shown in Figure 4.

Role-based access control has advantages such as increasing the flexibility of the system and facilitating the distributed management of the administrator. Such model can effectively solve the problems of system management complexity and security defects in access control and meanwhile design authority schemes that satisfy the requirements of roles by virtue of database interfaces. From this, such model can be regarded as a user + role + authority model.

In summary, comparing with the discretionary access control model and the mandatory access control model, the robe-based authority management model has remarkable advantages in terms of flexibility, security, and management modes; therefore, the role authority management model is selected as the system authority control model in this paper.

### 3.3. Design of Background Authority Functions

In the background architecture, the operation layer can facilitate the interaction of front page data and the related methods in the Dao layer can help with the processing of background data. Therefore, three types of background authority control functions are set here, namely, the Task Controller Function, the Project Controller Function, and the User Controller Function, so as to meet the requirements of different objects and subjects.

## 4. Design and Realization of Cloud Computing Based Role Authority Management Systems

### 4.1. Design of Cloud Computing Based Role Authority Management Systems

#### 4.1.1. Design of Database

After the authority control scheme is implemented, the background database side is needed to conduct tests. For MongoDB database belongs to distributed file storage NoSQL database, interactive orders can be employed for the goal of operating and accessing the database; meanwhile the storage structure is flexible and changeable, and therefore Spring Boot is utilized to facilitate the design and realization of MongoDB database. Besides, to guarantee the effectiveness of authority control, the view mode is utilized to measure the authority of user groups. Specifically speaking, directly see the authorities possessed by roles in every user group in the form of views and then operate in the page accordingly.

#### 4.1.2. Design of Database Background Architecture

The database background architecture is mainly composed of the Dao layer, the entity layer, and the operation layer. The entity layer here includes three entity classes, namely, the project, task, and user. The Dao layer enables operations such as deleting, adding, modifying, and querying of the database. The operation layer contains three related files, namely, the project, task, and user files. This layer can realize the front page data interaction; besides, it can also reasonably invoke the background data. And corresponding methods can be quickly found in the project class.

#### 4.1.3. Front Page Design and Parameter Passing

HTML/CSS/Javascript grammars are utilized to realize the development of front pages and the Boor Strap framework is introduced to obtain better front pages. To guarantee the effective interaction between the front-end and rear-end pages, Spring Boot is also utilized here. Besides, in returning JSON objects to the front end, the parameter passing employs the value of Ajax function in JQuery.

### 4.2. Realization of Cloud Computing Based Role Authority Management Systems

For the test system utilizes Docker during the deployment, the environment and dependence required by the project should be stored. After the image construction is completed, the whole set of service can be obtained by directly operating images. Everyone who wants to test the project effect can test on his own simply by laying Docker environment in his host to build images and thus to reduce the tedious test process for the test personnel.

#### 4.2.1. Configuration Environment

The hardware environment package of the cloud computing platform has multiple physical hosts matched with X86-64 chips. All the physical hosts carry Docker environments, chose Linux as the bottom layer operating system, and support 64-bit environment. Under the Ubuntu system, there are three steps in the configuration environment flow. First, examine the preparatory condition “uname-a” of the machine, upgrade the system kernel when it is found that the system kernel cannot meet the requirements of the design, and execute relevant installation operations only after the upgrading is completed. Meanwhile, to guarantee the normal installation of Curl order, add APT repository for assistance. Second, add GPG keys, renew the APT source, and then complete the installation of Docker software packages. Third, test the installation effect of Docker and execute “sudo docker info” order if the installation is determined to be normal. When no container or image is found in the order, the Docker environment is not completely installed, and we need to wait or reinstall it; otherwise, the installation of Docker environment is completed.

#### 4.2.2. Deployment File Writing

Docker-compose.yml and Dockerfile are the two core files necessary for the system deployment. In docker-compose.yml file, two types of images need to be written-in. The first is the images of the Spring Boot project. Spring Boot is a new framework developed by the Pivotal team to ease the difficulty of developing and building new Spring. Spring Boot is configured in a specific way rather than in traditional ways, avoiding manual configuration by developers. With this advantage, Spring Boot has been greatly promoted in the field of application development and has become the first choice of developers for system development. Spring Boot not only inherits the advantages of the Spring framework, but also optimizes the configuration, which further eases the difficulty of developing and building Spring applications. In addition, after the integration of a large number of frameworks, the problems of dependent package version conflict and application uncertainty are solved. The second is the images of MongoDB, the customization process of which is as follows: first, customize an nginx image and store the image in /usr/share/nginx/html/index.html file; second, input the From order and the RUN order; and third, execute the building action under the storage directory of Dockerfile. After the images are successfully built, it is necessary to set the context path and construct the image instructions, such as constructing the parameter instructions, defining the anonymous data volume instructions, constructing the port declaration instructions, and establishing the working directory instructions. The system can only operate normally after the two types of images are written-in, while in Dockerfile, the environment and dependence required by the project should be defined to realize the independent compilation of Docker.

#### 4.2.3. Project Deployment

Invoke and execute the “docker-compose up-d” order in the project, and then relevant images are obtained and the system is operated. The operation state of the containers can be directly checked through the “docker logs” order other than conducting secondary examination of the MongoDB containers because the information of MongoDB is integrated into the images of the Spring Boot project. When MongoDB fails to start, the start of the project will terminate. The specific working process of the project is as follows: first, monitor the user's URL request; second, analyze the user request and filter the URL content; third, complete the selection of back-end processing functions according to different parameters and request contents; fourth, call the back-end processing function and get response; and fifth, transfer the content that needs to be returned to the user and present it on the front page.

## 5. System Test

After the deployment is completed, the system is tested to verify the sound interaction between the cloud computing platform and the role authority management system. The interaction service is carried out at the entrance of the user access system, which enables users to visually learn about the real-time status of the project and the requests of users can be processed accordingly. Details are as shown in Table 2.

It can be seen that the cloud computing platform based role authority management system has satisfactory test results consistent with expected outputs as well as strong robustness. A part of the implementation interface of the cloud platform based role authority management system test is presented as shown in Figure 5.

It can be seen that the cloud computing platform based role authority management system has complete functions and can effectively disclose member information. The cloud computing platform and role authority management system have good interaction, which confirms the feasibility of the design of this paper.

## 6. Conclusion

This paper first gives an overview of the research in this field, analyzes authority control models, Docker, and other related technologies, determines the role authority control model based on the basic framework of Docker, and designs the role authority management system on this basis. Finally, the cloud computing platform is deployed, its interaction with the role authority management system is completed, and the core authority function is realized. Through the test, the function of the cloud computing platform based role authority management system is fully verified, and the feasibility of the model design is confirmed. With the continuous research and development as well as optimization of the model, the basic framework can completely replace traditional role authority management modes and then promote the development of role authority management.

Docker is a lightweight virtual technology with advantages of shorter deployment time and higher resource utilization rate than virtual machines. The deployment of the project on Docker enables the system to realize the purpose of multiple operations at one time, which greatly shortens development and testing time, improves work efficiency, and is highly practical. However, this technology also has some problems such as poor isolation performance and serious waste of storage resources, which affects the performance of the design architecture in this paper and indicates the direction for future research.

## Figures and Tables

**Figure 1:** Architecture of Docker.

**Figure 2:** Basic model architecture of the authority management system.

**Figure 3:** Model core structure.

**Figure 4:** Relation diagram of users, roles, and authorities.

**Figure 5:** A part of the implementation interface of the cloud computing platform based role authority management system.

**Table 1:** Decision rules.

		Object security level			
		A	B	C	D
Subject security level	A	I/Q	I	I	I
	B	Q	I/Q	I	I
	C	Q	Q	I/Q	I
	D	Q	Q	Q	I/Q

**Table 2:** System test results.

Item	Input/action	Expected output	Actual test result
Authority management	Users clicking the “Authority Management” button	Entering the role authority management interface	Test result consistent with the expected output
	Finding relevant content in the Find bar as needed	Displaying information found	Test result consistent with the expected output
	Clicking the “Modify” button	Displaying “Modify Authority”	Test result consistent with the expected output
Role management	Users clicking the “Role Management” button	Entering the role management interface	Test result consistent with the expected output
	Clicking the “Add” button	Displaying the user addition interface	Test result consistent with the expected output
	Clicking the “Modify” button	Displaying the user role modification interface	Test result consistent with the expected output
Node management	Clicking the “Query” button	Displaying all node definition information	Test result consistent with the expected output
	Clicking the “Delete” button	Displaying corresponding node to delete interface	Test result consistent with the expected output

## Data Availability

All the data contained in this study can be obtained by contacting the corresponding author. Readers can also inquire part of the original data and the results of data processing in this paper.
